# *Klebsiella pneumonia* and Its Antibiotic Resistance: A Bibliometric Analysis

**DOI:** 10.1155/2022/1668789

**Published:** 2022-06-06

**Authors:** Yanping Li, Suresh Kumar, Lihu Zhang, Hongjie Wu

**Affiliations:** ^1^Pharmacy Department, Jiangsu Vocational College of Medicine, 224005 Yancheng, Jiangsu Province, China; ^2^Post Graduate Centre, Management and Science University, University Drive, Off Persiaran Olahraga, Section 13, 40100 Selangor, Malaysia; ^3^Department of Diagnostic and Allied Health Science, Faculty of Health and Life Sciences, Management and Science University, Shah Alam, Malaysia; ^4^School of Electronic and Information Engineering, Suzhou University of Science and Technology, Suzhou, China

## Abstract

The rapid development of antibiotic resistance in K. pneumonia has led to a major concern. In order to analyze the hotspots and develop trends in this field through visual the analysis, this study used CiteSpace software to summarize the available data in the literature to provide insights. A total of 9366 research articles were retrieved from the Web of Science Core Collection, and the number of published papers is increasing year by year. The country with the most articles was the USA, followed by China and India. The institution with the highest number of publications was LERU. The author with the highest number of articles was Li. The journal with the highest citation rate was Antimicrobial Agents and Chemotherapy. In addition, based on keyword coword analysis and cited literature prominence analysis by CiteSpace, the current research focus in the field was therapy, CRKP, and resistance genes. This paper provides a new quantitative visualization way for the development of the field in the recent ten years. The results show global trends that researchers can use to determine future directions.

## 1. Introduction

*Klebsiella pneumonia*, belonging to the family *Enterobacteriaceae*, is a natural inhabitant of the gastrointestinal tract microbiome of healthy humans and animals [1]. It has a variety of antibiotic resistance mechanisms and is a common pathogen causing hospital-acquired surgical wound infections, digestive tract infections, and community-onset infections, which can cause outbreaks of nosocomial infection [2]. The global drug resistance rate of *K. pneumonia* has reached as high as 70%, and the infection-related fatality rate has also reached 40%~70% [3]. In recent years, multiple-drug resistance (MDR) *K. pneumonia* and *carbapenem-resistant Klebsiella pneumonia* (CRKP) have emerged as a major global public health problem.

In this study, we reviewed the literature on antibiotic resistance of *K. pneumonia* by bibliometrics [4]. This study is aimed at analyzing the trend of antibiotic resistance research of *K. pneumonia* in recent 10 years. According to data from the Web of Science Core Collection (WoSCC), the CiteSpace5.8.R3 software system was employed to display the detailed analysis based on visualization of the cooperative network of the countries, coauthors, and co-occurring keywords [5]. The method and results of this paper may provide potential prospects for the study of antibiotic resistance of *K. pneumonia* in the future.

## 2. Data Collection and Methodology

The data from 2012 to 2021 (10 years) were from WoSCC on April 13, 2022, to reduce bias incurred by database updating. Search terms were used as follows: “(((((((TS=(Antibiotic resistance)) OR TS=(Antibiotic resistant)) OR TS=(Antimicrobial Resistance)) OR TS=(Antimicrobial Resistant)) OR TS=(Drug Resistance)) OR TS=(Drug Resistant)) AND ((TS=(Klebsiella pneumonia)) OR TS=(K. pneumonia)) AND (EDN==(“WOS.SCI”) AND DT==(“ARTICLE” OR “REVIEW”) AND LA==(“ENGLISH”)))” in Advanced Search. In addition to data collection, the CiteSpace 5.8.R3 (64-bit) software system was also used to show the detailed data analysis. All records such as titles, abstracts, and references are exported to CiteSpace for subsequent analysis.

## 3. Results and Discussion

### 3.1. Publication Characteristics

The Web of Science Core Collection (WoSCC) database shows 9366 publications that use our search terms, with 8398 articles and 968 reviews. In general, the number of papers published in recent years shows an upward trend, which indicates that the number of papers published in antibiotic resistance research in *K. pneumonia* is receiving more and more attention from researchers. Especially in the past three years, the number of publications has increased sharply, accounting for almost half of the total number of publications. Therefore, the analysis period of this study is from 2012 to 2021, and the research period is divided into one year.

### 3.2. Countries/Regions and Institutions Co-Operation Analysis

The distribution of studies on antibiotic resistance research in *K. pneumonia* in different countries can be understood by analyzing the country information according to the affiliation of the authors. Many institutions or universities from different countries around the world have contributed to this research field. Research papers from 178 countries have been published, and we have listed the top 10 most productive and influential countries and institutions in *K. pneumonia* antibiotic resistance research field, based on the total publications, citations, and *H*-index during 2012–2021 (Figure 1). As shown in Table 1, the USA and China ranked first and second, with 1,908 and 1,416 publications, accounting for 20.37% and 15.12% of the total, respectively, ahead of India (664 publications and 7.09%), which ranked third. In regard to institutions (Table 2), League of European Research Universities (LERU) is the most productive institution in the field of “antibiotic resistance research in *K. pneumonia*” contributing 521 papers and 18990 total citations. Udice French Research Universities (UFRU) and Egyptian Knowledge Bank (EKB) are ranked second and third in terms of the number of papers.

Besides the total number of publications, the *H*-index, which represents the cited influence of papers, was given in the tables, too. Sometimes, a high total number of publications or citation number alone does not ensure a high *H*-index. Therefore, some scientists prefer to use the *H*-index to rank top countries (institutions), because this bibliometric indicator can more fully evaluate the impact of research [4].

In our case, in terms of “most productive countries,” the USA topped the *H*-index by a wide margin. However, in regard to prolific institutions, LERU is the most prolific institution with an *H*-index value of 65. We also analyzed the results using the CtieSpace 5.8.R3 to visually show the most productive countries (institutions) and their connections to each other (Figures 2 and 3). Meanwhile, to highlight the attention of core countries (regions) and relevant academic institutions in this field, the VOSviewer 1.6.18 and Scimago Graphica 1.0.17 software were used for analysis [6].

### 3.3. Authors' Coanalysis

Among the top 10 authors with publications, four are from China, three from the USA, two from Australia, and one from France, respectively, as shown in Table 3. Li of Monash University, Australia, tops the list with 87 publications. Bonomo from the USA and Wang from China ranked second and third, with 84 and 81 publications, respectively. On *H*-index, Bonomo (34) and Paterson (29) rank the top two, showing the absolute advantages and influence of these authors on antibiotic resistance research in K. pneumonia.

Generating a productive author collaboration network is shown in Figure 4. The size of the circle indicates the number of papers the author has published, and the lines between the circles indicate the connections between the authors. The group of primary core authors is the most representative and provides centralized information. From the centrality analysis, Paterson (0.25) ranked the highest followed by Hsueh (0.15), Badal (0.09), and Bonomo (0.09), which reflect their emphasis on this field.

### 3.4. Journal Analysis

From 2012 to 2021, a total of 1301 journals worldwide published academic papers on antibiotic resistance research in *K. pneumonia*. Among them, the number of publications of the top 10 journals is more than 140, accounting for 28.25% of the total number of publications, as shown in Table 4. Antimicrobial Agents and Chemotherapy ranked first in terms of published research with 426 articles, accounting for 4.54% of total articles, followed by Frontiers in Microbiology and Journal of Antimicrobial Chemotherapy, and 364 and 303 papers were published, respectively, accounting for 3.88% and 3.23% of the total publications. These top two journals also ranked first and second in average citation per article and *H*-index, respectively. Among the 10 journals, one is in Q1 subregion, and eight are in Q2 subregion with impact factors ranging from 3.0 to 5.7, among which, Journal of Antimicrobial Chemotherapy has the highest impact factor.

### 3.5. Keyword Analysis

#### 3.5.1. Coword Analysis

Through keyword coword analysis, research topics and hotspots can be analyzed, and the transition of research frontiers in a certain knowledge field can be monitored [7]. We used Citespace software to identify keywords from selected papers. At this stage, keywords with similar meanings were combined, such as “antibiotic resistance,” “antimicrobial resistance,” and “drug resistance.” Table 5 shows the top 10 keywords for frequency and centrality in this field over the past 10 years. We also developed networks for the analysis in Figure 5. It can be seen that the top five keywords of co-occurrence were *Klebsiella pneumonia*, antibiotic resistance, *Escherichia coli*, *Enterobacteriaceae*, and infection. In order of centrality, the top five keywords were biological activity (0.17), synergy (0.14), penetration (0.14), antimicrobial peptide (0.12), and high prevalence (0.12). Centrality refers to the ratio of the shortest path that passes through a certain point and connects the two points to the total number of shortest path lines between the two points, which is used to describe the importance of a node. The larger the value is, the more influential the node is in the key position in the network [8].

#### 3.5.2. Clustering Analysis

Keyword clustering analysis can cluster similar points together and identify clusters that represent relevant research areas. We use CiteSpace to summarize the clustering of the keyword timeline map. Cluster size is the number of terms contained in each cluster. CiteSpace gives cluster ID 0 to the largest cluster, cluster ID 1 to the second largest, and so on. As shown in Figure 6, the main research directions can be classified as follows: #0 whole genome sequencing, #1 antibacterial activity, #2polymyxin b, #3 identification, #4 combination therapy, #5 virulence, #6 drug resistance, #7 United States, #8 bactericidal activity, #9 mortality, #10 sequence, #11 liver abscess, #12 mgrb, #13 Escherichia coli, and # 14 carbapenem resistance: these clusters can summarize the development of antibiotic resistance research in *K. pneumonia* and reveal the current research hotspots.

### 3.6. Keyword and Reference Burst Detection

Keyword burst detection refers to a significant increase in the frequency of keywords in a short period of time. If we understand the studies with high attention in this period, we can judge the hot topics and frontiers of research in the field accordingly. Keyword burst detection of antibiotic resistance research in 10 years in *K. pneumonia* is shown in Figure 7(a). Sorted by emergence time, it can be seen that the research frontier is whole genome sequencing, activation, phage therapy, gut microbiota, and care associated infection. To some extent, this result represents the trend of the future research.

According to Figure 7(b), it can be seen that in the past 10 years that the research hotspot changes and advances the process of antibiotic resistance research in *K. pneumonia*. Depending on the burst strength, the first *t* papers are reviewed from two high-level journals: Lancet Infections Diseases and Clinical Microbiology Reviews [9–12]. The article with the strongest burst strength was published in Lancet Infect Dis in 2010, which reported a new antibiotic resistance mechanism of a new type of carbapenem resistance gene designated blaNDM-1 [13]. Another three papers show that the heat continues to this day. Two of them are reviews about *K. pneumonia* [14–17]. Another article was published in PNAS in 2015 which sequenced the genomes of 300 diverse *K. pneumonia* and performed a pan-genome-wide association study (PGWAS) to look for associations between gene profiles associated with virulence and antibiotic resistance and the differing disease outcomes seen for *K. pneumonia* [18].

## 4. Conclusion

This paper provides a visual and comprehensive literature review of antibiotic resistance research in *K. pneumonia*. We examined the characteristics of publications, collaboration between countries, institutions, and authors, and co-occurrence analysis of journals and keywords. In the past 10 years, there have been 9366 journal articles related to this field, and the number of publications increased rapidly, which showed that scientists are paying increasing attention to this area. Antibiotic resistance in *K. pneumonia* has emerged as a significant threat to global public health problems [19].

We find several interesting keywords with high co-occurrence frequency through co-word analysis. According to recent research, carbapenem-resistant Klebsiella pneumonia (CRKP) has been paid much attention. Carbapenems have strong antibacterial activity and a wide antibacterial spectrum. Carbapenems are the preferred drugs for the treatment of serious Enterobacteriaceae bacterial infections [20]. However, the emergence and prevalence of CRKP pose a serious threat to patients with low immune function and have become an independent risk factor leading to the death of patients with nosocomial infections [21].

Drug efflux, biofilm formation, enzymatic inactivation of the drug, alteration of drug targets, and reduced permeability due to porin loss or modification are the major mechanisms conferring antibiotic resistance to *K. pneumonia* [22]. For combating antibiotic resistance in *K. pneumonia* infections, several therapies are currently being developed. Phage therapy, phytotherapy, photodynamic therapy, antimicrobial peptides, and nanoantibiotics are the potential of some alternatives.

Phages have low natural toxicity and high strain specificity. Due to the specificity of phages, their action is limited to the site of infection and can prevent the destruction of the inherent microbiome [23]. This reduces the development cost of phage therapy compared to antibiotics [24].

Additionally, we highlight the highly cited papers and reveal the research hotspots on antibiotic resistance research in *K. pneumonia*. This paper uses CiteSpace software to perform bibliometrics and visualization analysis on antibiotic resistance research in *K. pneumonia* data from the Web of Science database. This work presents direct and specific ways to describe existing information in different perspectives to the reader and can provide reference and reference for the relevant scientific research workers in the topic selection and development direction of the research.

## Figures and Tables

**Figure 1:** (a) Publication volume and growth trends in each year on antibiotic resistance research of K. pneumonia from 2012 to 2021. (b) Publication volume and growth trends of the top 10 countries/regions on antibiotic resistance research of K. pneumonia from 2012 to 2021. Bar chart reflects number of publications per year.

**Figure 2:** The cooperation network of productive countries.

**Figure 3:** The cooperation network of prolific institutions.

**Figure 4:** Collaborative network of productive authors.

**Figure 5:** Co-occurrence network of keywords in research papers.

**Figure 6:** (a) Clustered networks of keywords in research papers via CiteSpace. The top 15 largest clusters are shown. (b) Timeline view of the top 15 largest clusters. The horizontal axis represents the evolution time, and #0-#14 represent keywords.

**Figure 7:** (a) Keywords with the strongest burst strength. Keywords marked in red indicate that the keyword usage frequency increases suddenly during this period. Blue represents a period of relative unpopularity. (b) References with the strongest burst strength. References marked in red indicate that the keyword usage frequency increases suddenly during this period. Blue represents a period of relative unpopularity.

**Table 1:** Top 10 most productive and influential countries.

Rank	Countries/regions	Publications	Citations	Average citation per item	*H*-index
1	USA	1908	65125	34.13	109
2	China	1416	24047	16.98	58
3	India	664	12636	19.03	50
4	Italy	550	16284	29.61	58
5	UK	530	21504	40.57	64
6	France	511	17375	34	61
7	Brazil	424	6720	15.85	38
8	Spain	397	11076	27.9	49
9	Australia	366	14155	38.67	60
10	Germany	360	9481	26.34	50

**Table 2:** Top 10 most productive and influential institutions.

Rank	Institutions	Publications	Citations	Average citation per item	*H*-index
1	League of European Research Universities (LERU)	521	18990	36.45	65
2	Udice French Research Universities (UFRU)	261	12201	46.75	51
3	Egyptian Knowledge Bank (EKB)	225	3633	16.15	30
4	Institut National de la Sante et de la Recherche Medicale (INSERM)	218	8951	41.06	41
5	Zhejiang University	197	7449	37.81	34
6	Assistance Publique Hopitaux Paris	171	8307	48.58	42
7	Universite de Paris	145	4532	31.26	33
8	US Department of Veterans Affairs	143	7162	50.08	44
9	Veterans Health Administration (VHA)	142	7059	49.71	44
10	Monash University	133	3825	28.76	33

**Table 3:** Top 10 authors in terms of publications.

Rank	Author	Publications	Citations	Average citation per item	*H*-index
1	Li (Australia)	87	2593	29.8	28
2	Bonomo (USA)	84	4852	57.76	34
3	Wang (China)	81	4608	56.89	21
4	Rolain (France)	75	2763	36.84	22
5	Chen (USA)	56	2077	37.09	24
6	Hsueh (China)	55	1642	29.85	23
7	Paterson (Australia)	55	4173	75.87	29
8	Liu (China)	53	562	10.6	13
9	Wang (China)	49	1045	21.33	16
10	Kreiswirth (USA)	47	2094	44.55	24

**Table 4:** Top 10 journals in terms of publication number.

Rank	Journal	Publications	Citations	Average citation per item	*H*-index	IF	JCR
1	Antimicrobial Agents and Chemotherapy	426	16731	39.27	69	5.191	Q2
2	Frontiers in Microbiology	364	8462	23.25	41	5.640	Q2
3	Journal of Antimicrobial Chemotherapy	303	8926	29.46	50	5.790	Q1
4	PLOS ONE	287	7119	24.8	46	3.240	Q2
5	Microbial Drug Resistance	250	2754	11.02	24	3.430	Q3
6	Infection and Drug Resistance	235	1869	7.95	21	4.003	Q2
7	Journal of Global Antimicrobial Resistance	225	1912	8.5	21	4.035	Q2
8	International Journal of Antimicrobial gents	222	5724	25.78	39	5.283	Q2
9	Antibiotics Basel	189	1226	6.49	17	4.639	Q2
10	BMC Infectious Diseases	145	2500	17.24	29	3.090	Q3

**Table 5:** Top 10 high-frequency keywords related to antibiotic resistance research in *K. pneumonia.*

Number	Freq.	Keyword
1	4345	Klebsiella pneumonia
2	4105	Antibiotic resistance
3	2791	Escherichia coli
4	1526	Enterobacteriaceae
5	1295	Infection
6	1107	Epidemiology
7	995	Pseudomonas aeruginosa
8	895	Prevalence
9	886	Risk factor
10	864	Emergence

## Data Availability

All data generated or analyzed during this study are included in this published article. Other data may be requested through the corresponding author.
